# Comprehensive Multiomics Analysis Reveals Potential Diagnostic and Prognostic Biomarkers in Adrenal Cortical Carcinoma

**DOI:** 10.1155/2022/2465598

**Published:** 2022-08-09

**Authors:** Xiunan Li, Jiayi Li, Leizuo Zhao, Zicheng Wang, Peizhi Zhang, Yingkun Xu, Guangzhen Wu

**Affiliations:** ^1^Department of Urology, The First Affiliated Hospital of Dalian Medical University, Dalian 116011, China; ^2^School of Business, Hanyang University, Seoul 15588, Republic of Korea; ^3^Department of Urology, Shandong Provincial Hospital, Cheeloo College of Medicine, Shandong University, Jinan 250021, China; ^4^Department of Urology, Dongying People's Hospital, Dongying 257000, China; ^5^Department of Urology, Shandong Provincial Hospital Affiliated to Shandong First Medical University, Jinan 250021, China; ^6^Department of Breast and Thyroid Surgery, The First Affiliated Hospital of Chongqing Medical University, Chongqing 400042, China

## Abstract

Adrenal cortical carcinoma (ACC) is a severe malignant tumor with low early diagnosis rates and high mortality. In this study, we used a variety of bioinformatic analyses to find potential prognostic markers and therapeutic targets for ACC. Gene Expression Omnibus (GEO) and The Cancer Genome Atlas (TCGA) data sets were used to perform differential expressed analysis. WebGestalt was used to perform enrichment analysis, while String was used for protein-protein analysis. Our study first detected 28 up-regulation and 462 down-regulation differential expressed genes through the GEO and TCGA databases. Then, GO functional analysis, four pathway analyses (KEGG, REACTOME, PANTHER, and BIOCYC), and protein-protein interaction network were performed to identify these genes by WebGestalt tool and KOBAS website, as well as String database, respectively, and finalize 17 hub genes. After a series of analyses from GEPIA, including gene mutations, differential expression, and prognosis, we excluded one candidate unrelated to the prognosis of ACC and put the remaining genes into pathway analysis again. We screened out CCNB1 and NDC80 genes by three algorithms of Degree, MCC, and MNC. We subsequently performed genomic analysis using the TCGA and cBioPortal databases to better understand these two hub genes. Our data also showed that the CCNB1 and NDC80 genes might become ACC biomarkers for future clinical use.

## 1. Introduction

Adrenal cortical carcinoma (ACC) originates from the adrenal cortex and is a rare clinical malignant endocrine tumor [1], with a population incidence of 0.001‰ to 0.002‰ [2]. Still, it is also the most common primary malignant tumor of the adrenal gland [3] and is the second most common malignant tumor of the endocrine organ after thyroid cancer [4]. ACC can occur at any age, with two peaks in childhood and between 50 and 70, and is more common in women [5–7]. The clinical manifestations of ACC are diverse and prone to invasion and metastasis. Due to the low early diagnosis rate and high mortality, the survival period is generally less than three years [8], and the 5-year survival rate is only 10% to 20% [9], which greatly threatens the life and health of patients. There is currently no effective early diagnosis and late treatment for ACC, and complete surgical resection is the only possible cure for ACC [10–13]. Therefore, finding novel biomarkers for efficient screening in the early stages of ACC may be valuable for long-term survival.

It is also worth noting that adrenocortical adenocarcinomas have distinct gene expression profiles from adrenocortical adenomas. The most widely recognized gene at present is the gene IGF2. The expression of IGF2 in adrenocortical adenocarcinoma is higher than that in adrenocortical adenoma. However, the differential diagnosis of adrenocortical adenocarcinoma and adrenocortical adenoma cannot be accurately performed by only using IGF2 as an indicator [14–16]. In recent years, research on differential genetic screening of adrenal tumors has been on the ascendant. It has been reported that the combination of IGF2 and Ki-67 has high specificity and sensitivity in identifying benign and malignant adrenal cortical tumors [12, 14, 17]. Another study reported that the most differentially significant genes were TOP2A, IGF2, CCNB2, CDC2, CDC25C, and CDKN1C [18]. The correlation between the differential gene expression fold and the survival time of patients with adrenocortical adenocarcinoma has also been confirmed [19], so it is possible to judge the prognosis of patients according to the gene expression level. In addition, steroidogenic factor 1 (SF-1), another gene that plays an essential role in promoting the occurrence and development of adrenal tumors, is of great significance to the growth and migration of adrenal tumor cells. In vivo experiments have proved that overexpression of SF-1 promotes the proliferation and migration of adrenocortical adenocarcinoma cells [20]. In addition, multiple studies have also confirmed that SF-1 has a high value in the diagnosis of adrenocortical carcinoma and the prognosis evaluation of patients [21–23], and it has been reported that SF-1 overexpression is associated with a low survival rate in patients with adrenocortical carcinoma. In addition, Snail is closely related to the metastasis and prognosis of adrenocortical carcinoma. The relevant research results show that more than 95% of the clinical stage III and IV adrenocortical carcinoma tumors have positive Snail expression [24]; ER-negative expression adrenal cortical carcinoma patients have a lower 5-year survival rate than those with ER-positive expression and have a greater chance of distant metastasis [25, 26]. In addition, the simultaneous high expression of BUB1B and PINK1 in tumor tissue may indicate a good prognosis in patients [27]. Therefore, the study of these differential gene expression profiles through bioinformatics analysis plays a crucial role in understanding the pathogenesis of adrenocortical adenocarcinoma and the molecular signaling pathways involved [28].

We first downloaded raw data from GEO and TCGA databases in this study to obtain differentially expressed genes (DEGs) in ACC. Then, we performed gene ontology, pathway enrichment analysis, and protein-protein interaction (PPI) network. GEPIA was adopted to observe these genes' mutations, differential expression, and prognostic characteristics. Besides, TCGA and cBioPortal were used to determine the distribution in pan cancers, pathway enrichment, the features in pathological parameters, and the relationship with other genes. We attempted to seek specific hub genes that may serve as influential biomarkers for ACC.

## 2. Materials and Methods

### 2.1. GEO Database

GEO is a gene expression database created and maintained by the National Center for Biotechnology Information NCBI. The database was built in 2000 and contains high-throughput gene expression data from research institutions worldwide. In this study, GEO database (http://www.ncbi.nlm.nih.gov/geo/) [29] was used for gene expression data sets between ACC tissues and normal tissues. Then, we further evaluated the complete information about the relevant data sets. Finally, in line with the Affymetrix Human Genome (GPL570) platform, two data sets (GSE19750 and GSE10927) were chosen for subsequent analysis. The GSE19507 data set contained 44 ACC and 4 normal samples [30, 31], and the GSE10927 data set included 33 ACC and 10 normal samples [32].

### 2.2. Differential Expression Analysis

R language was used to analyze GEO data and drew volcano maps and heat maps, and these two data sets were employed to get differential expressed genes (DEGs). |Log2FC|>1, *P*-value <0.05 was considered the cutoff criterion. Besides, we put on these data to cross with TCGA data [33]. Then, an online tool, Bioinformatics & Evolutionary Genomics, was used to draw the Venn diagram for up-regulated and down-regulated DEGs (http://bioinformatics.psb.ugent.be/webtools/Venn/) [34].

### 2.3. Gene Ontology and Pathway Enrichment Analysis

The up-regulated and down-regulated DEGs were integrated into the WEB-based Gene Set Analysis Toolkit (webgestalt) (http://www.webgestalt.org/) [35] for Gene Ontology (GO) functional annotation enrichment analysis. Furthermore, we performed KEGG pathway analysis for DEGs through the ClueGO plugin in Cytoscape software [36]. The KEGG [37], REACTOME [38], PANTHER [39], and BIOCYC [40] pathways were downloaded from the KOBAS website [41]. A *P*-value of <0.05 was considered statistically significant.

### 2.4. Protein-Protein Interaction (PPI) Network and Identification of Hub Genes

String database is a database that can be used to search for interactions between known and predicted proteins. In addition to generating beautiful protein-protein-interaction (PPI) maps of these proteins, an analysis of imported proteins is also provided. In this study, PPI network between DEGs was built by String database (http://stringdb.org/) [42]. First, entered the DEGs into the database and set the confidence score ≥0.7. Then, removed unlinked DEGs and arranged the remaining DEGs protein interaction data and photos. The data acquired by String website was substituted into the Cytoscape software and the hub genes were captured through the cytoHubba plugin. Afterward, the top 20 genes were collected by three algorithms of Degree, MCC, and MNC [43]. The Venn diagram of these hub genes was gathered using the online tool Bioinformatics & Evolutionary Genomics.

### 2.5. Gene Expression Analysis and Survival Analysis

GEPIA (http://gepia.cancerpku.cn/detail.php) [44] is a newly developed interactive web server for analyzing RNA sequencing expression data of 9736 tumors and 8587 normal samples in TCGA and GTEX projects. Based on GEPIA database, we checked the differences in hub gene expression between ACC and normal tissues. The predictive value of these genes in ACC was analyzed using the GEPIA database, and the cutoff value was set to 50%. The website automatically calculated the hazard ratio (HR) of 95% confidence interval and log-rank *P*-value and displayed it directly on the web page. *P*-value <0.05 was considered statistically significant.

### 2.6. TCGA and cBioPortal Data

The cancer genome map included sequencing and pathology data for 30 different cancers. The ACC (TCGA, Provisional) data set was selected, comprising data from 92 pathology reports. These DEGs were further conducted via cbioportal (http://www.cbioportal.org/index.do) [45]. The genomic analysis is covered with mutations and co-expression analysis. The co-expression and networking were calculated based on cbioportal's online instructions. *P*-value <0.05 was considered statistically significant.

### 2.7. Statistical Analysis

Statistical analyses of all data were performed using statistical software from all online databases. Statistical significance of differences between and among groups was assessed using the *t*-test. Statistical significance was set at ∗*P* < 0.05; ∗∗*P* < 0.01; and ∗∗∗*P* < 0.001.

## 3. Results

### 3.1. DEGs in ACC

In recent decades, differentially expressed genes have been the focus of research in the field of cancer research. DEGs in ACC were identified by examining two GEO data sets and TCGA data (Figures 1(a) and 1(b)). 490 DEGs consisting of 28 up-regulated genes and 462 down-regulated genes were finally obtained in our work (Figure 1(d), Table 1). In addition, to show the distribution of these DEGs on human chromosomes more specifically, we draw the corresponding heatmaps. The results showed that over-expressed genes were mainly distributed on chromosomes 5, 7, and 12 (Figure 1(c)).

### 3.2. Functional Enrichment of DEGs

GO functional enrichment analysis was performed on these DEGs, demonstrating that biological regulation, membrane, and protein binding of most genes were enriched in terms of BP, CC, and MF, respectively (Figures 2(a)–2(e)). Four pathway databases with KEGG, BIOCYE, REACTOME, and PANTHER revealed that ACC-related DEGs mainly concentrated on complement and coagulation cascades, metabolic pathways, malaria, ovarian steroidogenesis, and so on (Figures 3(a)–3(e)).

### 3.3. Identification of ACC-Associated Hub Gene

String database was applied to analyze the protein interactions of DEGs and make a PPI network (Figure 4(a)). The top 20 ACC-related hub genes were screened through three algorithms involving Degree, MCC, and MNC. After taking the intersection of these three data sets, 17 hub genes containing C3AR1, CCNB1, CDC20, CENPU, FOXM1, KIF4A, KIF11, KIF20A, MAD2L1, NCAPG, NDC80, NUF2, PBK, RACGAP1, RRM2, TOP2A, and TPX2 were collected for further study (Figures 4(b)–4(e)).

### 3.4. Hub Gene Expression and Prognosis in ACC

To better make out the 17 hub genes, we analyzed the mutations of 17 hub genes. The results showed that CENPU, FOXM1, and PBK had higher mutation rates accounting for 13%, 12%, and 11%, respectively (Figure 5(a)). Subsequently, we detected the expression of these hub genes in six tumors, including ACC, KICH, KIRC, KIRP, PAAD, and BLCA. CCNB1, MAD2L1, ACGAP1, and CENPU were significantly higher expressed in all six tumors (Figure 5(b)). Another discovery is that the expression analysis of these genes in ACC manifested that except for C3AR1, which was down-regulated in ACC, the other 16 genes were up-regulated in ACC (Figures 5(c) and 5(d)). In addition, we also found no significant correlation between C3AR1 and the prognosis of patients with ACC. Still, the rest of the hub genes had a great connection with an unfavorable prognosis (Figures 6(a)–6(q) and 7(a)–7(q)).

### 3.5. Functional Enrichment of Hub Genes

In cancer research, gene function enrichment analysis has become a routine method for high-throughput omics data analysis, which is of great significance for revealing biomedical molecular mechanisms. To better understand these hub genes' function, pathway enrichment analysis was performed on these 16 hub genes again, which suggested that hub genes were mainly associated with classical tumor-associated pathways, such as the P53 signaling pathway, and cell cycle-related signaling pathways (Figures 8(a)–8(d)).

### 3.6. Identification of Two ACC Core Genes CCNB1 and NDC80

By duplicating protein interaction analysis on these 16 hub genes and narrowing the core gene range, we derived two core genes, CCNB1 and NDC80 (Figure 9(a)). Then, we evaluated the expression of these two genes in pan cancers, and the consequences proved that these two genes were highly expressed in various tumors (Figures 9(b) and 10(a)). Further analysis suggested that the expression of CCNB1 and NDC80 would increase with disease progression. The high expression could also predict adverse outcomes in ACC patients but has little to do with gender (Figures 9(c) and 9(d) and 10(b) and 10(c)). To improve our knowledge about the functions of the core genes CCNB1 and NDC80, ten related proteins were retrieved by the String database (Figures 9(e) and 10(d)). Later, we discovered that CCNB1 and NDC80 participate in the same pathway, incorporated with cell cycle, progesterone-mediated oocyte maturation, HTLV-1 infection, and oocyte meiosis (Figures 11(a) and 11(b)). CCNB1 co-expressed with its related proteins CDK1, CDK2, CCNB2, PLK1, CDC20, CDCA8, ESPL1, and FZR1 (Figures 11(c)–11(j)) in ACC patients. Pathway analysis for NDC80 showed that NDC80 was associated with Cell Cycle (Figure 12(a)). It was worth mentioning that CCNB1 and NDC80 were consistently expressed in ACC (Figure 12(b)). Simultaneously, the expression of NDC80 also has collinearity with several proteins, like AURKB, BUB1, SPC25, and CENPE (Figures 12(c)–12(f)).

## 4. Discussion

In the past 20 years, molecular biology studies on ACC have made significant progress [46, 47], but this cancer's primary pathogenesis is still unclear. Moreover, recent epidemiological studies have shown that the incidence of ACC has increased yearly in the past 40 years, but the survival rate of patients has not improved [3]. As a highly malignant tumor, there is an urgent need to find effective diagnostic and prognostic targets for identifying early-stage patients, developing proper treatments, and improving ACC's poor prognosis. Therefore, using bioinformatics techniques to unravel the genomic properties of ACC at the molecular level is crucial for finding effective treatments and predicting patient survival and relapse risk, and there have been several successful cases of bioinformatics used in cancer research [48–51].

Our research selected GSE10927 (10 normal and 33 ACC tissues) and GSE19750 (4 normal and 44 ACC tissues) from the GEO database. After analyzing R language, these results were cross-correlated with data from TCGA, and 28 up-regulated and 462 down-regulated DEGs were enrolled for our study. Then, we carried out GO functional analysis and pathway analysis (KEGG, REACTOME, PANTHER, and BIOCYC) using WebGestalt and KOBAS websites to learn these candidates' gene function and regulatory process. Moreover, PPI network analysis was used to search for the hub genes through String database, and 17 dominant genes were considered. In addition, the cBioPortal database helped investigate the mutations in these genes. The GEPIA website was applied to assess the extent of differential expression, overall survival (OS), and disease-free survival (DFS). After excluding genes unrelated to ACC's prognosis, we repeated pathway analysis on the remaining genes and acquired two target genes by three different algorithms. Eventually, we demonstrated that CCNB1 and NDC80 were associated with ACC's diagnosis and prognosis and could be considered vital biomarkers for future clinical use.

CCNB1, also known as Cyclin B1, is essential for controlling cell cycle during the G2/M (mitosis) transition [52]. Our results showed that the expression of CCNB1 was elevated in many cancers compared to normal cases, such as esophageal cancer, gastric cancer, colorectal cancer, liver cancer, and breast cancer [53–56]. CCNB1 was positively correlated with the stage of ACC. As the degree of disease increased, the expression of this gene also increased. This denoted that CCNB1 can distinguish the severity of this cancer. Ten genes (ESPL1, CDK2, CDK1, ANAPC4, FZR1, PLK1, CDC27, CDC20, CCNB2, and ANAPC10) refer to 4 pathways (P53 signaling pathway, cell cycle, progesterone-mediated oocyte maturation, and oocyte meiosis) connected with CCNB1 were filtered out by our results. CCNB2 can compensate for CCNB1 in oocyte meiosis [57] and works consistently in ACC. CCNB1 and CDK1 were co-expressed in ACC, and this action was also acknowledged in breast cancer susceptibility, progression, and survival of Chinese women [58]. Lohberger et al. proposed that CCNB1 and CDK1/2 are involved in the G2/M cell cycle checkpoint, providing an inner relationship between CCNB1 and CDK family [59]. The combination of CCNB1 and CDC20 high expression could predict the poor prognosis of liver cancer [60], similar to what we got in ACC. In a word, CCNB1 was involved in the process of ACC disease progression and occupied the central position of several pathways, implying that it could become a potential gene for further study.

NDC80 is required for chromosome segregation and spindle checkpoint activity [61]. It could affect the growth of hepatocellular carcinoma [62] and promote proliferation and metastasis of colon cancer [62]. In our study, the expression of NDC80 was much higher in ACC stage 4 than in stage 1-3 but had nothing to do with gender. NDC80 was mainly centralized in cell cycle pathways and had protein interaction with CASC5, SPC25, AURKB, SPC24, NUF2, BUB1, ZWINT, CENPE, BUB1B, and MAD2L1. We should pay attention to whether NDC80 and CCNB1 had a co-expression in ACC, prompting that the combined detection of these two genes can improve the diagnostic rate of ACC. NDC80 could also be a promising marker to identify ACC and estimate the prognosis of this cancer.

## 5. Conclusions

Based on a series of bioinformatics analyses, our study concluded that CCNB1 and NDC80 are particularly relevant for the high risk and poor prognosis of ACC in theory, suggesting that these two genes can be beneficial for proper diagnosis and treatment of this disease. However, more efforts should be invested in clinical experiments to learn these genes' biological functions and pathological evolution in ACC.

## Figures and Tables

**Figure 1:** The process of identifying DEGs in ACC. (a–b) Volcano maps based on GSE10927 and GSE19750 data sets. (c) Schematic representation of differentially expressed genes on chromosomes. (d) Venn diagram based on DEGs in GSE10927, GSE19750, and TCGA data.

**Figure 2:** GO analysis was performed for DEGs in ACC. (a–c) Histograms show the results of GO analysis. (d–e) Hierarchical plots show the results of the GO analysis.

**Figure 3:** Pathway enrichment analysis was performed for DEGs in ACC. (a) Interaction plot showing the results of pathway enrichment analysis. (b–e) Bubble plots show KEGG, BIOCYC, REACTOME, and PANTHER pathway enrichment analysis results.

**Figure 4:** Protein-protein interaction analysis and screening of hub genes of DEGs. (a) The protein-protein interaction network of these DEGs molecules. (b) Top 20 hub genes screened by Degree algorithm. (c) Top 20 hub genes screened by MCC algorithm. (d) Top 20 hub genes screened by MNC algorithm. (e) A Venn diagram is drawn based on the hub genes obtained by Degree, MCC, and MNC algorithms.

**Figure 5:** Overall variation and mRNA expression of 17 hub genes in urological tumors. (a) Overall variation of 17 hub genes in ACC. (b) Expression of 17 central genes in urologic tumors. (c–d) mRNA differential expression of 17 hub genes in ACC.

**Figure 6:** Overall survival analysis. (a–q) Survival graphs showing the overall survival of these 17 hub genes in ACC, in order of C3AR1, CCNB1, CDC20, CENPU, FOXM1, KIF4A, KIF11, KIF20A, MAD2L1, NCAPG, NDC80, NUF2, PBK, RACGAP1, RRM2, TOP2A, and TPX2.

**Figure 7:** Disease-free survival analysis. (a–q) Survival graphs show the disease-free survival of these 17 hub genes in ACC, followed by C3AR1, CCNB1, CDC20, CENPU, FOXM1, KIF4A, KIF11, KIF20A, MAD2L1, NCAPG, NDC80, NUF2, PBK, RACGAP1, RRM2, TOP2A, and TPX2.

**Figure 8:** After removing the C3AR1 gene with no prognostic significance in ACC, pathway enrichment analysis was performed in ACC for the remaining 16 hub genes. (a) KEGG pathway. (b) BIOCYC pathway. (c) REACTOME pathway. (d) PANTHER pathway.

**Figure 9:** In-depth exploration of the biological value of the core gene CCNB1. (a) Venn diagram showing the identification of the core genes CCNB1 and NDC80. (b) mRNA expression of CCNB1 in pan-cancer. (c) mRNA expression of CCNB1 in different stages of ACC. The *P*-value between stage 1 and stage 4 is 2.2252E-04. (d) The effect of CCNB1 mRNA expression level and patient gender on the overall survival of ACC patients. (e) PPI map between CCNB1 and the ten most closely related CCNB1 protein molecules.

**Figure 10:** In-depth exploration of the biological value of the core gene NDC80. (a) mRNA expression of NDC80 in pan-cancer. (b) mRNA expression of NDC80 in different stages of ACC. The *P*-value between stage 1 and stage 4 is 5.7562E-03. (c) The effect of NDC80 mRNA expression level and patient gender on the overall survival of ACC patients. (d) PPI map between NDC80 and the ten most closely related NDC80 protein molecules.

**Figure 11:** Functional and co-expression analysis of CCNB1. (a–b) Pathway enrichment analysis of CCNB1. (c–j) Co-expression analysis of CCNB1 and related genes.

**Figure 12:** Functional and co-expression analysis of NDC80. (a) Pathway enrichment analysis of NDC80. (b–f) Co-expression analysis of NDC80 and related genes.

**Table 1:** 490 DEGs were identified from TCGA and GEO data sets, including 28 up-regulated and 285 down-regulated genes in ACC compared with normal tissues.

DEGs	Genes name
Up-regulated genes (*n* =28)	GGH TPX2, CCNB1, PLA2G1B, ANLN, MND1, FOXM1, KIF11, RACGAP1, CENPH, RRM2, TOP2A, ZNF367, CENPU, APOBEC3B, GPX8, MAD2L1, GAS2L3, KIF4A, KIF20A, CENPK, PDE8B, CDC20, NDC80, PBK, NUF2, NCAPG, ESM1

Down-regulated genes (*n* =462)	CLMP, FSTL1, MMP2, RALYL, NR4A2, SERPINF1, SUGCT, SLCO2B1, TEK, NEFH, GYPC, LINC00924, EMILIN1, ID1, CELA1, IGSF11, SLC9A3R1, FHL1, IRX3, IFITM10, BTK, SYTL5, USP9Y, AQP11, ZBED6CL, FAM49A, HOXA5, TAC1, HOTAIRM1, EPB41L3, TSTD1, ALAS1, DAAM2, SMOC2, MAN1A1, NKAIN1, CSDC2, LRRC32, EMB, AXL, SHE, TCEAL2, IL10, ALOX5AP, FMO3, ABCA6, NBEA, DDX3Y, MCOLN3, SLC16A4, MC2R, WISP1, BRE, SRPX, ZNF204P, ADAP2, EIF1AY, LRRN4CL, RARRES1, CLEC5A, MARCO, TIMP4, KCNMB4, C9orf3, AOX1, CYR61, TYMP, GGT5, APOC1, FLVCR2, DLGAP1-AS1, CHRDL1, LAMA2, C1QC, CD55, PLN, RERG, PLTP, MRPL33, PON1, DNASE1L3, RNASE2, ERMP1, SLC47A1, ABCB1, THBD, CHKB, TH, MAP3K8, SPON1, PLA2G4A, ABCC3, EDNRB, EGFLAM, DPYS, ADAMTSL2, C7, S100A8, NPY5R, ITGAM, FOSL2, SKAP1, CCR1, HTR2B, PYGL, HIBCH, COL4A4, SPOCK2, GPR34, CORO1A, EFEMP2, AEBP1, JAM2, RASD1, CYP11B1, GPRASP1, CDKN1C, TXLNGY, IL33, GPX3, NOV, GPM6B, AMT, HSD11B1, KCNJ5, ACOX2, ERN1, PTH1R, PHYHD1, NXPH1, DAPL1, NPC1, PARM1, MS4A14, FBLN5, FIBIN, MUM1L1, IGF1, CERK, SUSD2, CSF3R, SCUBE3, SERPINB9, GATA6, MRAP, SERPING1, PDZRN3, MFAP5, COLEC11, MGST1, STON1, PAX8-AS1, CEBPD, NGFR, NEDD4L, PDGFD, SGK1, KRT8, NFKBIZ, SLC25A34, PLCXD3, RAMP3, TINAGL1, S100A16, TNFSF13, EFEMP1, LUM, C1S, FCGRT, NGEF, PLAT, SRPX2, IGFBP6, SLC37A2, AKAP12, HSD3B2, APOD, AKR1B1, MAPK13, TNFRSF14, ARFGAP3, CYP17A1, IL4R, OLFML3, FXYD1, FCER1G, C11orf96, RSPO3, CCDC159, SREBF1, C2orf40, KCNJ8, CFD, C1QTNF1, AS3MT, PITPNM1, ACTR3C, ANKS1A, SYNPO2, ALPK3, NR2F1, EPHA2, FAM150B, RASGRP2, PTPRB, PNMAL2, ECM1, DNALI1, STEAP4, LILRA2, B4GALT6, TTC39C, STX11, ACO1, SFRP4, FAM166B, DNAJC12, RXFP1, RAPGEF4, EPHX2, CCDC68, DUOX1, ACSM5, PLIN1, SULT1E1, RARRES2, ADAMTS1, TMEM173, GLUL, RASSF2, AVPR1A, TCIRG1, NPR2, ZEB2, PYY2, FMO2, MEST, SCNN1A, FAM65C, IGFBP4, NANOS1, RETSAT, OLFML1, NCF4, SIRPB2, KCNK3, FGR, HEPH, PHYHIP, C5AR1, APOE, GKN1, CRHBP, THRB, MCOLN2, LONRF2, SORBS2, MTMR6, PACSIN3, OMD, TCF21, SLA, KLF2, ACADVL, SLC16A2, SIGLEC1, MGP, ECHDC3, CPA4, GIMAP6, MYC, GPM6A, STARD8, FNDC4, F13A1, GIPC2, OGN, SLC44A3, CXCL2, STAB1, THBS1, AMDHD1, TMEM200C, SYBU, FILIP1L, SCN7A, MCF2, PDGFRA, SLC27A2, CPE, DHRS1, DCN, CYB5A, C1orf162, CYP4B1, COL12A1, HOPX, EIF2D, ARHGEF10L, ZDHHC2, ST6GALNAC5, FCGR2B, MAP3K5, ACRC, CRYAB, PARVA, C8orf4, SLC40A1, CORO2B, ITGA8, IL1RL1, MS4A6A, IFITM2, BHMT2, FRMD6, GBP2, ATP1B2, LINC01314, USP53, G0S2, C10orf10, SHC3, CTGF, CD163, DPT, PTGDS, IGSF10, NKD2, CXCL12, ALDH1A1, CARTPT, PPAP2B, C1QB, CBLN4, BRINP2, IFI35, TLR4, ZNF185, C9orf24, TMOD1, LPAR1, ADAMTSL3, CRISPLD2, SELENBP1, FOSL1, CNTN6, S100A9, KLHL2, LRFN5, GLT8D2, CNN1, SIGLEC9, ALDH3A2, PLEKHO1, SLCO2A1, MEIS2, PRPS2, TLE2, ACSF2, HCK, CSRP1, MAP7, DGAT1, NPY1R, TPD52L1, SHISA8, GPR182, MRC1, IGFBP5, PTGER4, KCNQ1, ANGPTL1, IGSF21, CD14, TRIP6, KLHDC8A, EMCN, SLC27A6, ISLR, DKK3, MS4A4A, MYLK, ACSBG1, PID1, ADORA3, RAI2, GCKR, FBP1, ST3GAL4-AS1, VASN, ALDH1A3, DOK2, SELM, BOC, TMEM61, PRELP, WFDC1, CYBRD1, PLEKHA6, HGF, CYP1B1, VAMP8, C1R, SQRDL, TRIM22, CD33, NR1H3, AADAC, CACHD1, GSTA4, ABCA1, C3AR1, CFH, CHGA, SLC1A5, MT1M, TNNC1, DUSP26, FBLN1, SLC16A9, CD248, LMOD1, ZRANB1, LAT2, VSIG4, THRSP, FMO1, ARNTL, CCL2, FAM179A, RBKS, TAGLN, KCNK2, MOXD1, MFAP4, DLG2, ARHGAP9, PLEK2, RBP4, S100A4, PROK1, ACKR1, CREG1, FNDC5, PCDH10, NEXN, GATA5, BICC1, INMT, ITM2A, MPDZ, TMEM220, ADH1B, CAB39L, FSTL3, FCN3, GATA6-AS1, GAREM, KDM5D, VIPR1, GRAMD3, HCLS1

## Data Availability

The data used to support the findings of this study are available from the corresponding author upon request.

## Abbreviations

ACC: Adrenocortical carcinoma
TCGA: The Cancer Genome Atlas
GEO: Gene Expression Omnibus
GEPIA: Gene expression profiling interactive analysis
C3AR1: Complement C3a receptor 1
CCNB1: Cyclin B1
CDC20: Cell division cycle 20
CENPU: Centromere protein U
FOXM1: Forkhead box M1
KIF4A: Kinesin family member 4A
KIF11: Kinesin family member 11
KIF20A: Kinesin family member 20A
MAD2L1: Mitotic arrest deficient 2 like 1
NCAPG: Non-SMC condensin I complex subunit G
NDC80: NDC80 kinetochore complex component
NUF2: NUF2 component of NDC80 kinetochore complex
PBK: PDZ binding kinase
RACGAP1: Rac GTPase activating protein 1
RRM2: Ribonucleotide reductase regulatory subunit M2
TOP2A: DNA topoisomerase II alpha
TPX2: TPX2 microtubule nucleation factor
KICH: Kidney chromophobe
KIRC: Kidney renal clear cell carcinoma
KIRP: Kidney renal papillary cell carcinoma
PAAD: Pancreatic adenocarcinoma
BLCA: Bladder urothelial carcinoma
ESPL1: Extra spindle pole bodies like 1, separase
CDK2: Cyclin-dependent kinase 2
CDK1: Cyclin-dependent kinase 1
ANAPC4: Anaphase promoting complex subunit 4
FZR1: Fizzy and cell division cycle 20 related 1
PLK1: Polo-like kinase 1
CDC27: Cell division cycle 27
CCNB2: Cyclin B2
ANAPC10: Anaphase promoting complex subunit 10
SPC25: SPC25 component of NDC80 kinetochore complex
AURKB: Aurora kinase B
SPC24: SPC24 component of NDC80 kinetochore complex
BUB1: BUB1 mitotic checkpoint serine/threonine kinase
ZWINT: ZW10 interacting kinetochore protein
CENPE: Centromere protein E
BUB1B: BUB1 mitotic checkpoint serine/threonine kinase B.
